The article "Synthesis of new 2-amino-1,3,4-oxadiazole derivatives with anti-salmonella typhi activity evaluation" was published in 2020. Journal: BMC Chem.

# Synthesis of new 2-amino-1,3,4-oxadiazole derivatives with *anti*-*salmonella typhi* activity evaluation

**DOI:** 10.1186/s13065-020-00682-6

**Published:** 2020-04-20

**Authors:** Eid E. Salama

**Affiliations:** 1 Chemistry Department, College of Science and Arts, Jouf University, Qurayyat, Kingdom of Saudi Arabia; 2 Chemistry Department, Faculty of Science, Suez Canal University, Ismailia, Egypt

**Keywords:** Oxadiazole, Acid chloride, Aromatic thiol, Amino acid, Anti-salmonella typhi

## Abstract

Reaction of phenyl acetic acid derivatives with thiosemicarbazide in the presence of POCl_3_ afforded 5-(4-bromobenzyl)-1,3,4-oxadiazole-2-amine **1** and 5-(3-nitrophenyl)-1,3,4-oxadiazole -2-amine **2**. Acylation of the amino group of oxadiazoles **1** and **2** with some acid chlorides such as methyl 4-(chlorocarbonyl) benzoate, 3-nitrobenzoyl chloride, 4-methoxy-benzoyl chloride, 4-isobutylbenzoyl chloride and chloroacetyl chloride yielded the acylated compounds **3**–**8**. Cyclization of acetamides **7** and **8** by reaction with ammonium thiocyanate gave the thiazolidinones **9** and **10**. Coupling of chloroacetamide **7** with two mercaptothiazoles gave coupled heterocyclic derivatives **11** and **12**. Coupling of amino-oxadiazole **1** with *N*-Boc-glycine and *N*-Boc-phenylalanine lead to the formation of **16** and **17** respectively. All compounds were screened for their antibacterial activity against *Salmonella typhi* where compounds **3**, **4**, **10**, **11** and **15** showed significant activity. Structures of the new synthesized compounds were confirmed using the spectral analysis such as IR, ^1^H NMR and ^13^C NMR and mass spectrometry.

## Introduction

Oxadiazoles derivatives represent an important class of heterocyclic compounds with broad spectrum of biological activity. Oxadiazoles have been reported to possess anti-inflammatory [1, 2], anti-HIV [3], antibacterial [4, 5], anticonvulsant activities [6], antimalarial [7], herbicidal [8], antianxiety [9], insecticidal [10], antitubercular [11], antiviral [12], antifungal [13, 14], anti-HBV [15], anticancer [16], analgesic [17].

Typhoid is actually an infection as a result of *Salmonella typhi* which causes symptoms [18]. Symptoms can vary from gentle to extreme and in most cases, start 6 to 30 days soon after exposure. Frequently there is a progressive beginning of a very high fever more than several days. Weaknesses, abdominal pain, constipation, and migraines also commonly happen [19]. Diarrhea is uncommon, and vomiting is not usually severe. Some people develop a skin rash with rose-colored spots [20, 21].

*Salmonella enterica* subsp. enterica is a subspecies of *Salmonella enterica*, the rod-shaped, flagellated, aerobic, Gram-negative bacterium. Many of the pathogenic serovars of the *S. enterica* species are in this subspecies, including that responsible for typhoid [22].

Herein, we synthesized about seventeen new oxadiazole derivatives and screen them against *Salmonella typhi* to find new leads.

## Results and discussion

4-Bromophenylacetic acid and 3-nitrobenzoic acid was allowed to react with semicarbazide in presence of phosphorus oxychloride followed by basification of product with potassium hydroxide to give 5-(4-bromobenzyl)-1,3,4-oxadiazole-2-amine **1** and 5-(3-nitrophenyl)-1,3,4-oxadiazole-2-amine (**2**).

Oxadiazole **1** or **2** were acylated by methyl-4-(chlorocarbonyl)-benzoate, 3-nitrobenzoyl chloride, 4-methoxybenzoyl chloride or 4-tert-butylbenzoyl chloride in presence of triethylamine to give *N*-acyl derivatives **3**–**6** (Scheme 1).

**Scheme 1:** Synthesis of *N*-substituted oxadiazole derivatives

Oxadiazole **1** and **2** were reacted with chloroacetyl chloride in presence potassium carbonate to give *N*-(5-(4-bromobenzyl)-1,3,4-oxadiazole-2-yl)-2-chloroacetamide **7** and *N*-(5-(3-nitrophenyl)-1,3,4-oxadiazol-2-yl)-2-chloroacetamide **8** respectively. Refluxing **7** and **8** with ammonium thiocyanate in ethanol gave 2-[{(5-(4-bromobenzyl)-[1, 3, 4] oxadiazol -2-yl}-imino]-1,3-Thiazolidin-4-one **9** and 2-[{5-(3-nitrophenyl)-[1, 3, 4]-oxadiazol-2-yl}-imino]-1,3-thiazolidin-4-one **10**. Acyl chloride **7** reacted with benzo[d]thiazole-2-thiol and 4,5-dihydro-thiazole-2-thiol to give compounds **11**–**12** (Scheme 2).

**Scheme 2:** Cyclization and thiolation of chloroacetamide oxadiazole derivatives

Oxadiazole **1** was refluxed with 3-chlorophenyl isocyanate in ethanol to afford 1-(5-(4-bromobenzyl)-1,3,4-oxadiazole-2-yl)-3-(3-chlorophenyl)urea **13**.

Coupling of oxadiazole **1** with *N*-protected amino acids such as *N*-Boc glycine and *N*-Boc phenylalanine gave *tert*-butyl-(5-(4-bromobenzyl)-1,3,4-oxadiazole-2-ylcarbamoyl)-methyl-carbamate **14** and *tert*-butyl-1-(5-(4-bromobenzyl)-1,3,4-oxadiazol-2-ylcarbamoyl)-2-phenylethyl-carbamate **15** respectively. Deprotection of **14** and **15** was carried out by reaction with trifluoroacetic acid in presence of anisol to give *N*-(5-(4-bromobenzyl)-1,3,4-oxadiazol-2-yl)-2-amino acetamide **16** and *N*-(5-(4-bromobenzyl)-1,3,4- oxadiazol-2-yl)-2-amino-3-phenyl propanamide **17** as salts (Scheme 3).

**Scheme 3:** Reaction of oxadiazole 1 with chlorophenyl isocyanate, glycine and phenylalanine

## Structure confirmation

Structure **1** has confirmed by infrared spectra which showed well defined bands attributable for *ν*_C=N_ at 1610 cm^−1^ and *ν*_NH2_ at 3310–3400 cm^−1^. The 4-bromophenyl ring revealed two doublets at d 7.215 and 7.497 ppm. Characteristic singlet of methylene group appeared at 4.097 ppm and the amino group was found as singlet at 7.006 ppm. ^13^C-NMR of 1 revealed the presence two carbon of oxadiazole ring around 169.0 and 157.3 ppm, carbons of 4-bromophenyl appeared around 137.9 and 120.5 ppm whereas, the methylene carbon appeared at 35.2 ppm. The ^1^H-NMR of 5-(3-nitrophenyl)-1,3,4-oxadiazole-2-amine **2** amino group at 7.622 ppm. ^13^C NMR spectrum revealed the two oxadiazole carbons at 169.0 and 164.7 ppm. ^1^H-NMR spectrum for compounds **3**–**6** showed NH signal appeared around 12.00 ppm. Infrared spectra showed well-defined bands attributed to *ν*_NH_ at 3200–3400 cm^−1^. ^1^H NMR of **7** and **8** showed new signal for CH_2_ around 4.00 ppm. ^13^C NMR of **9** and **10** spectrum showed signal for Carbon of methylene group at signal at 35.4 ppm. Structure of **12** deduced from ^1^H NMR which displayed two triplet signals at 3.43 and 4.05 ppm for two methylene groups.

Structure of compound **13** was assigned from the characteristic two singlet’s for two NH groups at 9.52 and 12.23 ppm. The methylene protons found at 4.26 ppm. Infrared spectra showed well-defined bands attributable for *ν*_C=O_ at 1653.80 cm^−1^ and *ν*_NH_ at 3369.59 cm^−1^. Structure of compound **14** and **15** confirmed from ^1^H NMR which revealed the nine protons of *tert*-butyl group at 1.34 ppm, two methylene groups at 3.81 and 4.31 ppm, two NH groups at 7.16 and 12.80 ppm. ^1^H NMR of 16 and 17 proved the removal *N*-Boc group and formation of **16** and **17** moreover, F^19^ NMR showed signal around 73.84 ppm indicating the presence of fluoride.

### Antibacterial activity

The novel seventeen compounds were screened for their antibacterial activity against gram negative bacteria *Salmonella typhi* at three concentrations i.e. 1000, 100 and 10 ppm using ditch dilution method. The test organism was a 2-h culture of *Salmonella typhi* incubated and grown in peptone-water medium (temperature 37 °C). DMF was used as solvent control which did not show any zone of inhibition. Muller-Hilton agar medium was used as culture medium. The culture plates were incubated at 37 °C for 24 h. Antibacterial activity was determined by measuring the diameter of the inhibition zone. The results are given in Table 1. Compounds **3**, **4**, **10**, **11** and **15** displayed greater antibacterial activity against *Salmonella typhi*. Especially Compounds **10** and **11** exhibited the broadest spectrum activity in this series due to the heterocyclic ring of the imine and sulfide. Whereas, compounds **2**, **5**, **6**, **8**, **9**, **12** and **16** showed moderately activity. Resistance of bacteria to these synthesized compounds could be associated to alteration of the bacterial protein targeted by compounds, enzymatic degradation of the synthesized compounds, or change in the membrane permeability to them.

**Table 1:** The activity of the tested compounds against *Salmonella typhi*

Compound	*S. typhi*	Compound	*S. typhi*
1	+	10	+++
2	++	11	+++
3	+++	12	++
4	+++	13	+
5	++	14	+
6	++	15	+++
7	–	16	++
8	++	17	+
9	++		

+++strongly active, ++moderately active, +weakly active range, –inactive

### Experimental

All melting points were uncorrected, performed on a MEL-TEMP II. Melting point apparatus. Microanalysis was performed by micro analytical laboratory, Cairo University, Egypt. Infrared spectra were recorded (ν in cm^−1^) with pye Unicam SP 1200 spectrophotometer and using KBr Wafer technique. Mass spectra were measured with a Thermo Scientific LTQ Linear Ion Trap. Nuclear magnetic resonance spectra (^1^H NMR, ^13^C NMR) were recorded (δ in ppm) on Bruker (300 MH_z_) spectrometer. The purity of the synthesized compounds was checked by TLC on glass coated plates in the laboratory with silica gel GF 254 type, 60 mesh, size 50–250.

### Synthesis of 5-(4-bromobenzyl)-1,3,4-oxadiazole-2-amine (**1**) and 5-(3-nitrophenyl)-1,3,4-oxadiazole-2-amine (**2**)

The mixture of 4-bromophenyl acetic acid and/or 3-nitro benzoic acid (1 mol) and semicarbazide (0.455 g, 1 mol) were dissolved in 3 mL of phosphorus oxychloride and refluxed for 45 min. The reaction was cooled to room temperature then 3 mL of water was added carefully. The mixture was refluxed for 4 h, filtered on hot and the solid washed by warm water and the filtrate was basified with saturated potassium hydroxide. The precipitate was filtered off and recrystallised from ethanol.

#### 5-(4-Bromobenzyl)-1,3,4-oxadiazole-2-amine **1**

Yield 65%; mp: 200–202 °C; IR (KBr) cm^−1^: 3310–3400 (NH_2_), 1610 (C=N); ^1^H NMR (300 MHz, DMSO-d_6_, δ ppm): 4.097 (s, 2H,–CH_2_–), 7.006 (s, 2H, –NH_2_), 7.215 (d, 2H, J = 8.18 Hz), 7.4971 (d, 2H, J = 8.079 Hz); ^13^C NMR (DMSO-d_6_, δ ppm): (169.0, 157.3, 137.9, 132.0, 131.4, 120.5, 35.2); ESI–MS: 252 (100%), 254 (98%). Anal. Calcd. For C_9_H_8_BrN_3_O (252.99): C, 42.54; H, 3.17; N, 16.54. Found C, 42.51; H, 3.12; N, 16.50.

#### 5-(3-Nitrophenyl)-1,3,4-oxadiazole-2-amine **2**

Yield 60%, mp: 236–238 °C. IR (KBr) cm^−1^: 3330–3410 (NH_2_), 1610 (C=N); ^1^H NMR (300 MHz, DMSO-d_6_, δ ppm): 7.71–8.45 (m, 4H, ArH), 7.622 (s, 2H, –NH_2_); ^13^C NMR (DMSO-d_6_, δ ppm): (169.0, 164.7, 148.5, 133.7, 130.6, 127.4, 122.4, 121.6); ESI–MS: 206 (100%). Anal. Calcd. For (206.04): C, 46.61; H, 2.93; N, 27.18. Found: C, 46.57; H, 2.89; N, 27.14.

### Reaction of oxadiazoles 1 and 2 with acid chlorides derivatives

To a solution of 5-(4-bromobenzyl)-1,3,4-oxadiazole-2-amine **1** and/or 5-(3-nitrophenyl)-1,3,4-oxadiazole-2-amine **2** (0.5 mol) in methylene chloride (20 mL) containing triethylamine (0.069 mL, 0.5 mol), methyl-4-(chlorocarbonyl)-benzoate, 3-nitro-benzoyl chloride, 4-methoxybenzoyl chloride and/or 4-tert-butylbenzoyl chloride (0.5 mol) were added. The reaction mixture was stirred continuing at room temperature for overnight. The solvent was evaporated under vaccum and the residue was extracted by EtOAc and washed by NH_4_Cl, dil HCl(1 N)/water and brain (NaCl). The product formed after evaporation was recrystallized from ethanol.

#### Methyl-4-(5-(4-bromobenzyl)-1,3,4-oxadiazole-2-ylcarbamoyl)benzoate **3**

Yield 70%, mp: 281–283 °C. 3430 (NH), 3057 (aromatic C–H), 1683 (C=O), 1605, 1551, 1440 (C=N and C=C). ^1^H NMR (300 MHz, DMSO-d_6_, δ ppm): 3.8622 (s, 3H, –CH_3_), 4.3417 (s, 2H, –CH_2_), 7.2866 (d, J = 8.199 Hz, 2H), 7.5122 (d, J = 8.202 Hz, 2H), 8.0324 (d, J = 8.3310 Hz, 2H), 8.1431 (d, J = 8.253 Hz, 2H), 12.6132 (s, 1H, –NH); ^13^C NMR (DMSO-d_6_, δ ppm): (166.1, 165.6, 163.3, 161.4, 137.7, 137.1, 133.2, 132.1, 131.6, 129.7, 129.2, 120.6, 53.0, 34.8); ESI–MS: 415 (100%), 417 (98%). Anal. Calcd. For C_18_H_14_BrN_3_O_4_ (415.02): C, 51.94; H, 3.39; N, 10.10. Found: C, 51.91; H, 3.36; N, 10.07.

#### N-(5-(4-bromobenzyl)-1,3,4-oxadiazole-2-yl)-3-nitrobenzamide **4**

Yield 75%, mp: 294–296 °C; IR (KBr) cm^−1^: 3420 (NH), 1610 (C=N), 1670 (C=O); ^1^H NMR (300 MHz, DMSO-d_6_, δ ppm): 4.336 (s, 2H,–CH_2_), 7.274 (d, J = 8.24 Hz, 2H), 7.4900 (d, J = 8.1 Hz, 2H), 7.7516 (t, 1H), 8.389–8.414 (dd, 2H), 8.866 (s, 1H), 12.3157 (s, 1H, –NH); ^13^C NMR (DMSO-d_6_, δ ppm): (165.6, 163.3, 161.4, 148.2, 137.4, 135.1, 134.0, 132.0, 131.5, 130.7, 127.5, 123.6, 120.7, 34.7); ESI–MS: 402 (100%), 404 (98%). Anal. Calcd. For C_16_H_11_BrN_4_O_4_ (402): C, 47.66; H, 2.75; N, 13.90. Found: C, 47.63; H, 2.73; N, 13.86.

#### N-(5-(4-bromobenzyl)-1,3,4-oxadiazole-2-yl)-4-methoxybenzamide **5**

Yield 70%, mp: 281–283 °C; IR (KBr) cm^−1^: 3260 (NH), 1635 (C=N), 1673 (C=O); ^1^H NMR (300 MHz, DMSO-d_6_, δ ppm): 3.3447 (s, 3H, –CH_3_), 4.3263 (s, 2H, –CH_2_), 7.0336 (d, J = 8.61 Hz, 2H), 7.2713 (d, J = 7.95 Hz, 2H), 7.4913 (d, J = 8.13 Hz, 2H), 8.0581 (d, J = 8.85 Hz, 2H), 12.7404 (s, 1H, –NH); ^13^C NMR (DMSO-d_6_, δ ppm): (164.7, 163.4, 160.2, 137.6, 132.0, 131.5, 130.9, 123.9, 120.6, 114.3, 56.0, 34.6); ESI–MS: 387 (100%), 389 (98%). Anal. Calcd. For C_17_H_14_BrN_3_O_3_ (387.02): C,52.60; H, 3.63; N, 10.82. Found: C, 52.57; H, 3.59; N, 10.78.

#### 4-tert-Butyl-N-(5-(3-nitrophenyl)-1,3,4-oxadiazole-2-yl)benzamide **6**

Yield 65%, mp: 290–291 °C; IR (KBr) cm^−1^: 3320 (NH), 1640 (C=N), 1674 (C=O); ^1^H NMR (300 MHz, DMSO-d_6_, δ ppm): 1.29 (s, 9H, –(CH_3_)_3_), 7.55–8.69 (m, 8H, ArH), 11.53 (s, 1H, –NH); ^13^C NMR (DMSO-d_6_, δ ppm): (165.6, 160.8, 160.4, 156.8, 148.8, 133.8, 132.2, 131.7, 128.9, 126.0, 125.3, 121.3, 35.4, 31.3); ESI–MS: 366 (100%). Anal. Calcd. For C_19_H_18_N_4_O_4_ (366.13): C, 62.29; H, 4.95; N, 15.29. Found: C, 62.24; H, 4.90; N, 15.24.

### Reaction of oxadiazole-2-amine 1 and 2 with chloroacetyl chloride

To a solution of 5-(4-bromobenzyl)-1,3,4-oxadiazole-2-amine **1** and/or 5-(3-nitro-phenyl)-1,3,4-oxadiazole-2-amine **2** (1 mol) and potassium carbonate (0.69 g, mmole) in Dimethylformamide (11 mL), chloroacetyl chloride (0.075 mL, 1 mol) was added dropwise. The mixture was stirred well at room temperature for 4 h. Left to cool then pour the reaction mixture carefully onto crushed ice/water. The solid product that formed was filtered, washed with water three times, dried and recrystallised from ethanol.

#### N-(5-(4-bromobenzyl)-1,3,4-oxadiazole-2-yl)-2-chloroacetamide **7**

Yield 80%, mp: 233–234 °C; IR (KBr) cm^−1^: 3419 (NH), 1653 (C=O); ^1^H NMR (300 MHz, DMSO-d_6_, δ ppm): 4.2554 (s, 2H, –CH_2_), 4.3675 (s, 2H, –CH_2_), 7.2493 (d, J = 8.31 Hz, 2H), 7.4971 (d, J = 8.34 Hz, 2H), 12.8013 (s, 1H, –NH); ^13^C NMR (DMSO-d_6_, δ ppm): (165.8, 163.9, 159.1, 137.5, 132.1, 131.6, 120.7, 42.8, 34.6); ESI–MS: 328 (77), 330 (100). Anal. Calcd. For C_11_H_9_BrClN_3_O_2_ (328.96): C, 39.97; H, 2.74; N, 12.71. Found: C, 39.92; H, 2.70; N, 12.67.

#### *N*-(5-(3-nitrophenyl)-1,3,4-oxadiazole-2-yl)-2-chloroacetamide **8**

Yield 65%, mp: 168–170 °C; IR (KBr) cm^−1^: 3419 (NH), 1653 (C=N); ^1^H NMR (300 MHz, DMSO-d_6_, δ ppm): 4.45 (s, 2H, –CH_2_), 7.73–8.61 (m, 4H, ArH), 12.91 (s, 1H, –NH); ^13^C NMR (DMSO-d_6_, δ ppm): (166.0, 160.4, 159.4, 148.6, 133.7, 131.5, 131.2, 125.3, 120.4, 42.7); ESI–MS: 282 (100%). Anal. Calcd. For C_10_H_7_ClN_4_O_4 (_282.02): C, 42.49; H, 2.50; N, 19.82. Found: C, 42.45; H, 2.45; N, 19.78.

### Synthesis of thiazolidin-4-ones **9** and **10**

Compound **7** and/or **8** (7 mmol) and ammonium thiocyanate (15 mmol) in ethanol 35 mL were refluxed for 3 h, the reaction mixture was left overnight. The obtained precipitate was filtered off, dried and recrystallised from ethanol–water to yield compounds **9** and **10**.

#### 2-(5-(4-bromobenzyl)-1,3,4-oxadiazol-2-ylimino)thiazolidin-4-one **9**

Yield 75%, mp: 261–263 °C; IR (KBr) cm^−1^: 3215 (NH), 1641 (C=N), 1672 (C=O); ^1^H NMR (300 MHz, DMSO-d_6_, δ ppm): 4.3292 (s, 2H, –CH_2_), 4.0470 (s, 2H, –CH_2_), 7.2614 (d, J = 8.31 Hz, 2H), 7.5054 (d, J = 8.31 Hz, 2H), 12.2460 (s, 1H, –NH); ^13^C NMR (DMSO-d_6_, δ ppm): (174.4, 170.9, 166.09, 166.05, 137.3, 132.0, 131.5, 120.7, 36.0, 35.4); ESI–MS: 351 (100), 353 (98). Anal. Calcd. For C_12_H_9_BrN_4_O_2_S (351.96): C, 40.81; H, 2.57; N, 15.86. Found: C, 40.76; H, 2.52; N, 15.81.

#### 2-(5-(3-nitrophenyl)-1,3,4-oxadiazole-2-ylimino)1,3-thiazolidin-4-one **10**

Yield 60%, mp: 107–110 °C; IR (KBr) cm^−1^: 3230 (NH), 1645 (C=N), 1674 (C=O); ^1^H NMR (300 MHz, DMSO-d_6_, δ ppm): 4.10 (s, 2H, –CH_2_), 7.77–8.62 (m, 4H, ArH), 12.4 (bs, 1H, –NH); ^13^C NMR (DMSO-d_6_, δ ppm): (173.6, 171.2, 164.1, 163.4, 148.3, 133.3, 130.1, 127.6, 123.5, 122.7, 32.4); ESI–MS: 305 (100%). Anal. Calcd. For C_11_H_7_N_5_O_4_S (305.02): C, 43.28; H, 2.31; N, 22.94. Found: C, 43.24; H, 2.27; N, 22.89.

### Reaction of **7** with aromatic thiols

To a solution of *N*-(5-(4-bromobenzyl)-1,3,4-oxadiazole-2-yl)-2-chloroacetamide **7** (0.314 g, 1 mol) in dimethylformamide (20 mL), containing diisopropylethylamine (0.17 mL, 1 mol) under nitrogen, benzo[d]thiazole-2-thiol and/or 4,5-Dihydrothiazole-2-thiol (1 mol) was added. The reaction mixture was stirred well at room temperature for 4 h. Then the reaction mixture was poured into crushed ice/water, the formed solid was filtered, washed by water and recrystallised from chloroform.

#### N-(5-(4-bromobenzyl)-1,3,4-oxadiazole-2-yl)-2-(benzo[d]thiazol-2-ylthio)-acetamide **11**

Yield 60%, mp: 240–242 °C; IR (KBr) cm^−1^: 3310 (NH), 1640 (C=N), 1680 (C=O); ^1^H NMR (300 MHz, DMSO-d_6_, δ ppm): 4.42 (s, 2H, –CH_2_CO), 4.22 (s, 2H, –CH_2_), 7.22–7.97 (m, 8H, ArH), 11.86 (s, 1H, –NH); ^13^C NMR (DMSO-d_6_, δ ppm): (170,2, 168.6, 166.3, 166.8, 154.1, 135.7, 133.7, 132.9, 131.2, 125.1, 124.6, 122.3, 121.5, 120.4, 39.2, 32.1); ESI–MS: 461 (100%), 459 (98%). Anal. Calcd. For C_18_H_13_BrN_4_O_2_S_2_ (459.97): C, 46.86; H, 2.84; N, 12.14. Found: C, 46.81; H, 2.80; N, 12.11.

#### 2-(4,5-dihydrothiazol-2-ylthio)-N-(5-(4-bromo-benzyl)-1,3,4-oxadiazole-2-yl)-acetamide **12**

Yield 60%, mp: 259–260 °C; IR (KBr) cm^−1^: 3290 (NH), 1644 (C=N), 1685 (C=O); ^1^H NMR (300 MHz, DMSO-d_6_, δ ppm): 3.4321 (t, 2H, –CH_2_), 4.0512 (t, 2H, –CH_2_), 4.0783 (s, 2H, –CH_2_), 4.3213 (s, 2H, –CH_2_), 7.2637 (d, J = 8.33 Hz, 2H), 7.5053 (d, J = 8.35 Hz, 2H), 12.4894 (s, H, –NH); ^13^C NMR (DMSO-d_6_, δ ppm): (171.1, 167.9, 165.8, 163.1, 133.1, 132.4, 131.6, 121.3, 68.1, 35.2, 31.4, 30.1). ESI–MS: 413 (100%), 411 (96%). Anal. Calcd. For C_14_H_13_BrN_4_O_2_S_2_. (411.97): C, 40.68; H, 3.17; N, 13.56. Found: C, 40.62; H, 3.13; N, 13.52.

### Synthesis of 1-(5-(4-bromobenzyl)-1,3,4-oxadiazole-2-yl)-3-(3-chloro-phenyl)urea **13**

To a solution of 5-(4-bromobenzyl)-1,3,4-oxadiazole-2-amine **1** (0.15 g, 0.5 mol) in ethanol (15 mL), 3-chlorophenyl isocyanate was added, the reaction mixture was refluxed for 6 h. The precipitate was filtered off and recrystallized from ethanol.

### *1*-*(5*-*(4*-*bromobenzyl)*-*1,3,4*-*oxadiazole*-*2*-*yl)*-*3*-*(3*-*chloro*-*phenyl)urea***13**

Yield 60%, mp: 178–180 °C; IR (KBr) cm^−1^: 3369.59 (NH), 1653.80 C=O (amide); ^1^H NMR (300 MHz, DMSO-d_6_, δ ppm): 4.26 (s, 2H, –CH_2_), 7.02–7.68 (8H Ar), 9.52 (s, 1H, –NH), 12.23 (s, H, –NH); ^13^C NMR (DMSO-d_6_, δ ppm): (161.9, 153.5, 140.9, 137.5, 133.7, 132.1, 131.6, 130.9, 122.8, 120.7, 118.5, 117.6, 34.9); ESI–MS: 405 (78%), 407 (100%). Anal. Calcd. For C_16_H_12_BrClN_4_O_2_ (405.98): C, 47.14; H, 2.97; N, 13.74. Found: C, 47.11; H, 2.92; N, 13.70.

### Reaction oxadiazole-2-amine **1** with amino acid

To a solution of 5-(4-bromobenzyl)-1,3,4-oxadiazole-2-amine **1** in methylene chloride (20 mL), (0.268 g, 1 mol) and/or *N*-(*tert*-butoxycarbonyl)glycine, *N*-(*tert*-butoxy-carbonyl)phenylalanine was added followed by addition of dimethyl-aminopyridine (DMAP) (0.0122 g, 0.1 mol). *N*,*N*’-dicyclohexyl-carbodiimid (0.206 g, 1.1 mol) was added to the reaction mixture. The mixture was stirred at 0 °C for 1 h and it continued overnight at room temperature. The reaction mixture filtered off and washed with methylene chloride. The filtrate evaporated under vacuum and the residue was purified by column chromatography (EtOAc: Hexane, 1:1). The solid formed after evaporation was recrystallised from ethanol.

#### tert-Butyl-(5-(4-bromobenzyl)-1,3,4-oxadiazole-2-ylcarbamoyl)methyl-carbamate **14**

Yield 60%, mp: 188–190 °C; IR (KBr) cm^−1^: 3425.8 (NH), 1667.3, 1700.5 (2C=O); ^1^H NMR (300 MHz, DMSO-d_6_, δ ppm): 1.3390 (s, 9H), 3.8112 (d, J = 5.8 Hz, 2H, –CH_2_), 4.3102 (s, 2H, –CH_2_), 7.1556 (s,1H, –NH), 7.2489 (d, J = 8.106 Hz, 2H), 7.4843 (d, J = 8.127 Hz, 2H), 12.8013 (s, 1H, –NH); ^13^C NMR (DMSO-d_6_, δ ppm): (169.4, 163.3, 159.3, 156.3, 137.6, 132.1, 131.5, 120.7, 78.7, 43.6, 34.6, 28.6); ESI–MS: 410 (57.7), 412 (56.9), 354 (98), 356 (100), 310 (50.7), 352 (50), 208 (59.2). Anal. Calcd. For C_16_H_19_BrN_4_O_4_ (410.06): C, 46.73; H, 4.66; N, 13.62. Found: C, 46.69; H, 4.61; N, 13.57.

#### tert-Butyl-1-(5-(4-bromobenzyl)-1,3,4-oxadiazole-2-ylcarbamoyl)-2-phenyl-ethylcarbamate **15**

Yield 60%, mp: 177–180 °C; IR (KBr) cm^−1^: 3250–3440 (NH), 1675, 1755 (2C=O); ^1^H NMR (300 MHz, CDCl_3_, δ ppm): 1.2341 (s, 9H), 3.8124 (d, 2H, –CH_2_), 4.2974 (s, 2H, –CH_2_), 4.7374 (s,1H, CH), 6.4417 (s,1H, –NH), 7.1605–7.4558 (m, 9H), 12.8013 (s, 1H, –NH); ^13^C NMR (300 MHz, CDCl_3_, δ ppm): (171.7, 163.5, 160.9, 155.5, 136.0, 135.4, 132.1, 130.5, 129.2, 128.6, 127.3, 121.6, 79.8, 56.8, 35.5, 37.8, 28.1); ESI–MS: 500 (61.7), 502 (64.7), 446 (100), 444 (94.6), 402 (51.8), 400 (48.1). Anal. Calcd. For C_23_H_25_BrN_4_O_4_ (500.11): C, 55.10; H, 5.03; N, 11.17. Found: C, 55.06; H, 4.97; N, 11.12.

### Deprotection of *N*-protected group in compound **14** and **15**

Protected compounds **14** and **15** (1 mol) in methylene chloride (3.75 mL) was stirred under nitrogen followed by cooling in an ice bath then trifluoroacetic acid (1.25 mL) was added dropwise for 10 min followed by 0.05 mL of anisole. The reaction mixture was stirred for 2 h. Then it evaporated under vaccum. The oil product was crushed by ether (30 mL) and formed solid was recrystallised from acetone.

#### N-(5-(4-bromobenzyl)-1,3,4-oxadiazole-2-yl)-2-aminoacetamide **16**

Yield 75%, mp: 270–272 °C; IR (KBr) cm^−1^: 3320 (NH), 1660 (C=O), 2950 (NH salt); ^1^H NMR (300 MHz, DMSO-d_6_, δ ppm): 3.8975 (s, 2H, –CH_2_), 4.3482 (s, 2H, –CH_2_), 7.2637 (d, J = 6.39 Hz, 2H), 7.5034 (d, J = 6.813 Hz, 2H), 9.34179 (s, 3H, –NH_3_), 12.5478 (s, 1H, –NH); ^13^C NMR (DMSO-d_6_, δ ppm): (166.2, 163.8, 158.7, 137.5, 132.1, 131.6, 120.7, 41.3, 34.6); F^19^ NMR (DMSO-d_6_, δ ppm): − 73.838 (F); ESI–MS: 310 (100), 312 (97.8). Anal. Calcd. For C_11_H_11_BrN_4_O_2_ (310.01): C, 42.46; H, 3.56; N, 18.01. Found: C, 42.41; H, 3.52; N, 17.96.

#### N-(5-(4-bromo-benzyl)-1,3,4-oxadiazole-2-yl)-2-amino-3-phenylpropanamide **17**

Yield 75%, mp: 263–265 °C; IR (KBr) cm^−1^: 3270 (NH), 1672 (C=O) 2970 (NH salt); ^1^H NMR (300 MHz, DMSO-d_6_, δ ppm) 3.7516 (s, 2H, –CH_2_), 4.1342 (s, 2H, –CH_2_), 4.8951 (t, 1H, CH), 8.6579 (s, 3H, –NH_3_), 7.1203–7.8542 (m, 9H), 12.8013 (s, 1H, –NH); ^13^C NMR (DMSO-d_6_, δ ppm): (168.1), 164.0, 158.8, 137.4, 134.8, 132.0, 131.5, 129.8, 129.0, 127.7, 120.7, 54.3, 39.0, 37.1); F^19^ NMR (DMSO-d_6_, δ ppm): − 73.934 (F); ESI–MS: 400 (95.4), 402 (100). Anal. Calcd. For C_18_H_17_BrN_4_O_2_ (400.05): C, 53.88; H, 4.27; N, 13.96. Found: C, 53.82; H, 4.21; N, 13.90.

## Conclusion

Seventeen new functionalized oxadiazole hits were synthesized and characterized. The new hits were evaluated for their biological activity against gram-negative bacteria *Salmonella typhi*, among synthesized **3**, **4**, **10**, **11** and **15** demonstrated strong activities which recommends them for further studies to be future leads.

## Data Availability

All data and material analyzed or generated during this investigation are included in this manuscript. The raw data can be requested from email of Eid: eidsalama2000@gmail.com.
